# Analysis of Surveying and Mapping Method of Landownership and Environmental Resources Confirmation Based on GPS Technology

**DOI:** 10.1155/2022/8417692

**Published:** 2022-08-31

**Authors:** Fanye Dai

**Affiliations:** Business School, University of Nottingham, Hubei, Jingzhou 434000, China

## Abstract

The establishment of the agricultural and forestry land management information system is predicated on the acquisition of spatial positioning data of agricultural and forestry land, i.e., the surveying and mapping of agricultural and forestry land. It also serves as the central component of the overall management information system. It is necessary to find solutions to the issues of large plot areas and far-reaching boundary lines in light of the current situation of land right confirmation. With its high efficiency, the use of GPS technology for land right confirmation can not only increase work productivity and speed up construction but also lower operating costs. The method of confirming landownership through surveying and mapping is studied in this paper using GPS technology. With respect to various land types, various classification methods have varying degrees of classification accuracy. This method is one of the three algorithms that classify green land, which includes grassland, cultivated land, and forest land; however, it does not clearly distinguish between forest land and grassland, with forest land having an average classification accuracy of 58.69 percent. The average accuracy of classifying forest land is 73.14 percent. The classification accuracy of forest land using this method is 88.45 percent, which is a relatively high percentage. It can be seen that this method is more accurate in identifying minute differences between ground objects. This is demonstrated by comparing the accuracy of forest land classification with that of other methods. A lot of surveying and mapping work has been done on the assumption that urban control networks have been established in many cities. The most ideal option is to combine GPS technology with high-precision photogrammetry.

## 1. Introduction

The confirmation of land right is the identification of the location, boundary address, ownership nature, right subject, and identity of the land. The measurement of landownership confirmation is the basic work for the standardization of landownership confirmation registration, the registration of landownership according to law, and the settlement of landownership disputes. It is one of the important foundations for the fine production of land in the current society. The cadastral control survey is based on the accuracy requirements of boundary points and cadastral map, and the number and level of existing control points in the visual survey space area and test area [1]. It is necessary to carry out relevant design planning in accordance with the basic measurement criteria and accuracy requirements, so as to better handle relevant measurement work. The acquisition of spatial positioning data of agricultural and forestry land, that is, the surveying and mapping of agricultural and forestry land, is the premise for the establishment of agricultural and forestry land management information system, and also the core of the whole management information system [2, 3]. The land surveying and mapping technology has experienced from the steel ruler combined with the scale measurement method, which is difficult to deal with arcs and broken lines, to the theodolite combined with steel ruler measurement method to solve irregular land, and then to the total station measurement method, which is convenient for application and does not need to be erected on the land. In the survey of landownership confirmation and registration, we are faced with the problems of a large parcel of land and long distance between boundary lines. If the total station is used to collect cadastral elements, the layout of its control network is highly required and difficult to achieve [4]. The main purpose of surveying and mapping for the confirmation and certification of rural contracted land is to effectively solve the problems of area calculation and graphic analysis in the process of certification. It is a basic work to establish the information system in the surveying and mapping method for the confirmation and certification of rural contracted land. However, at present, in China, generally speaking, agricultural and forestry land surveying and mapping and information acquisition are still at a relatively backward stage, and most areas are still at the original measurement level of tape measurement, manual calculation, and manual recording [5, 6]. The reason is that on the one hand, some measurement methods are not applicable to the measurement of agricultural and forestry land and that on the other hand, the new technology measurement equipment has the limitations of complex operation [7], difficult to use, and requiring professional operation. Therefore, in the surveying and mapping of agricultural and forestry land, there is an urgent need for the development and popularization of high-precision and easy-to-operate surveying and mapping equipment.

The purpose of land right confirmation is to ascertain the location, boundary, ownership type, and right subject of land resources. It is a crucial foundation for the development and management of land resources. The issues of a large plot area and a great distance between boundary lines must be resolved in light of the current situation regarding the confirmation of land rights, and various new technologies must be actively applied on the foundation of already existing technologies. Among them, the use of GPS technology for land right confirmation has a high efficiency, and it can be used to improve work efficiency, speed up construction, and lower operating costs [8]. The term “GPS technology” refers to both real-time differential GPS technology and real-time dynamic measurement technology based on carrier phase observation. GPS technology, which primarily consists of a mobile station, reference station receiver, and data link, represents a significant advancement in the field of surveying. Real-time dynamic differential positioning (RTDDP) technology such as GPS is primarily based on reference station and mobile station high-precision carrier phase observations [9, 10]. The reference station typically needs to have a GPS receiver that can continuously track visible satellites and use radio transmission equipment to send observation data in real time to the user observation station. In addition to receiving the satellite signal, the GPS receiver in the mobile station also receives data sent from the reference station through wireless receiving equipment [11]. The three-dimensional coordinates of the mobile station are then acquired and precisely positioned in accordance with the relative positioning.

With the continuous progress and development of social economy, the control area of the existing control network has been completely unable to meet the needs of all aspects at present. Some control points have suffered great damage, so at this time, we will continue to use positioning technology to strengthen and improve the existing control network as the first-level control network of the cadastral survey [12]. In the process of using GPS technology to measure the urban cadastral control network, it should be combined with the original control points. The GPS survey technology constructs a reasonable survey team according to the size of the operation area before the survey. Each team member will work together to ensure the completion of the measurement. The general situation measurement team consists of instrument operator, recorder, and navigator, which can be adjusted according to the actual situation. It is necessary to carry out relevant design planning according to the basic measurement criteria and accuracy requirements, so as to better handle the related measurement work using GPS technology to measure the urban cadastral basic control network. According to other methods of surveying boundary coordinates, mapping cadastral maps by aerial survey is the most important way of urban foundation survey in China at present. In many cities, urban control networks have usually been established, and a lot of surveying and mapping work has been done under this premise. It is the best choice to use high-precision photogrammetry technology under GPS technology.

The main innovations I put forward in this paper are as follows:

1. This paper constructs the composition model of GPS satellite signal. In order to ensure the accuracy of the survey results, the application of GPS technology in landownership survey must choose an area with an open field of vision and no cover in the air, which is convenient for the mobile station and the reference station to transmit the survey information through the GPS satellite signal composition model. Compared with other surveying technologies, GPS technology has greatly reduced the number of staff in practical application, and one person can complete the collection of land surveying information, which provides a basis for the development and management of land resources and promotes the expansion of the project schedule.
2. The advantages of GPS measurement are discussed. Land use survey is the main means to understand the characteristics and laws of land resources and to master the quantity, quality, and distribution pattern of land resources, and is the basic work to carry out land resources research. GPS is used to measure three-dimensional coordinate data. In practical application, two-dimensional images are generally used to display the geographic information of farmland. Because the requirement of measurement accuracy is far lower than that of professional surveying and mapping, and only the local area is measured, the simplified method is adopted for data calculation.

## 2. Related Work

The physical foundation of human production, daily life, and social progress is land. In order to support the reform of rural collective land, safeguard farmers' land rights and interests, and reduce the tension between rural people and their land, it is crucial to confirm the right to rural collective land, as well as to ascertain the status of that land's use and the division of ownership. The cadastral management system in China today is fundamentally different from the one in place prior to liberation. Land is owned by the working class throughout China's socialist nation. Establishing a cadastral management system will improve China's land resources planning and the protection of working people's property.

Zhao makes clear the land parcel, area, and location by carrying out right confirmation registration, which is conducive not only to the protection of cultivated land, but also to the formulation and implementation of a series of policies to strengthen agriculture and benefit agriculture. It is also helpful for the state to formulate modern agricultural development plans, issue policies and measures to promote land transfer, and guide the standardized transfer of land based on the registered data [13]. Sediyono and Windarni put forward the work of confirmation, registration, and certification of rural land contractual management right, which is based on the existing rural land contractual management account, contract, and certificate, to find out the area and spatial location of the contracted land, establish and improve the land contractual management right register, and properly solve the problems of inaccurate contracted land area, unclear four directions, unknown spatial location, imperfect register, etc. [14]. In his research paper, Wang briefly described several land survey methods in different periods and different technical means, and gave a bird's-eye view of the changes and development of some land survey methods in recent years: from the measurement method of steel ruler combined with scale, to the measurement method of warp gauge combined with steel ruler, to the total station measurement method, and finally mentioned the measurement method of total station combined with the digital soil measurement system [15]. Feng proposed that in the land right confirmation work, satellite images were generally used before. With the development of UAV technology, the images taken by UAVs have the advantages of high resolution, good image quality, stable received signals, and so on. They are relatively good data sources [16]. Hauser et al. proposed the role of stabilizing the rural land contract relationship. The two-tier management system based on household contract management and the combination of unification and decentralization is the basis of the party's rural policy. A solid land contracting relationship and a better understanding of the plots, areas, and spatial locations contracted by the common people will help consolidate the party's rural land contracting and management system [17]. Zheng and Di Rong proposed that when reviewing the development of surveying and mapping instruments in history and looking forward to the development trend of surveying and mapping instruments, they introduced in detail the real estate boundary survey in ancient Egypt, the magnetic compass in ancient China, and the ancient surveying and mapping method and instruments of “left line, right rule” in Dayu's flood control [18]. Wang et al. put forward that due to local protectionism, backward economy and technology, and other reasons, there are false and concealed rural collective land use data in some places, which makes it difficult for the state to master accurate rural collective land use data. This phenomenon seriously affects land management, interferes with the state's scientific planning and decision-making on rural collective land, and lays hidden dangers for rural economic development and social harmony [19]. Quan Fu proposed to directly calculate the three-dimensional coordinates of boundary points by automatically recording the height angle, horizontal angle, and oblique distance of each detail point on the field electronic notebook or handheld computer, then using the photographic mapping technology. Photogrammetry, also known as aerial photogrammetry, is to obtain the specific orientation of the target by following aerial photographs and measuring negatives [20]. Wang proposed that high-quality rural collective land use data are the basis for promoting national development and social progress, and the basis for ensuring the sustainable and healthy development of the national economy [21]. Octavia A proposed that the period of updating and changing the utilization of rural collective land is becoming shorter and shorter. In order to master the utilization status of rural collective land, strictly enforce the land use management system, and promote the reform of rural collective land, the state has made a major decision to carry out the confirmation of the rights of rural collective land [22].

Based on GPS technology, this paper studies the surveying and mapping method of landownership. From the perspective of rural collective landownership production units, it studies how to control the process of rural collective landownership data and check the spatial data results before warehousing, so as to improve the quality of rural collective landownership spatial data, and reduce the data errors and then smoothly warehousing. According to the requirements of rapid land area measurement and information management, GPS technology develops portable area measuring instruments and land management information system, and provides a scientific basis for agricultural production and planning management. This paper analyzes the main aspects of data inspection under GPS technology, and puts forward the basic ideas of automatic inspection for polygon overlap inspection, gap inspection, and duplicate line inspection, as well as line discount and boundary line less vertex inspection.

## 3. Method

### 3.1. Principle and Model of GPS Technology

A satellite navigation system with a medium-distance circular orbit is the global positioning system (GPS). For locations on the surface of the earth, the global positioning system (GPS) offers precise positioning, velocity measurement, and high-precision time standards. It is necessary to choose a location with an open field of vision and no cover in the air for the application of GPS technology in the land right confirmation survey in order to ensure the accuracy of survey results [23]. This will make it easier to transmit survey information between mobile stations and reference stations via the model made up of GPS satellite signals. GPS technology has significantly reduced the amount of staff needed in actual applications when compared to other survey technologies. Additionally, one person can finish the collection of land survey data, serve as the foundation for the development and management of land resources, and support the expansion of project progress. The carrier, ranging code, and data codes that make up the satellite signal are all produced using the same reference frequency, as are the other signal components.  Figure 1 depicts the GPS satellite signal's composition model.

The GPS workflow consists of four steps:

1. Selection and inspection of instruments when selecting receiving equipment; it is best to use dual-frequency or multifrequency receivers, and ensure the stability of the equipment. When selecting the base station receiving equipment, the equipment with the function of transmitting standard differential data shall be selected.
2. Selection of reference station in the process of GPS-RTK measurement; the accuracy of measurement directly depends on the quality of data transmission. Therefore, it is very important to select the location of the reference station. A good reference station can ensure the transmission quality of the data link [24].
3. Setting of reference station after the site of the reference station is selected; the receiver antenna shall be installed first. It can be installed at either a known point or an unknown point. The setting process of the reference station is basically similar to that of the static surveying and mapping, including centering, leveling, and measuring antenna height.
4. GPS survey in the land right confirmation survey; RTK survey is divided into three steps: the first step is to start the reference station. When the reference station is erected at a known point, the current WGS-84 coordinates are entered to start the reference station. If an unknown point is erected, the WGS-84 coordinates measured by single-point positioning shall be sent to the GPS host for startup.

GPS can realize a unique spatial information system. In terms of implementation and modeling, it has shown its unique characteristics and advantages. First, a receiver is set on the reference station, which is used as the reference station to observe the satellite, and the observed data and station information are transmitted to the mobile station.

GPS can uniformly geocode the vector data of the parcel information, and can associate the vector data with the relational data, so as to complete the display of the parcel location. The schematic diagram of the GPS satellite positioning principle is shown in Figure 2.

After the GPS radio signal is received by the user receiver, if the clock of the receiver is accurately synchronized with the satellite clock, the time from the GPS satellite to the GPS user receiver can be measured, and the time difference is the propagation time of the satellite signal in space.

(1) $$\begin{array}{c} \Delta t^{\prime }=t_{2}-t_{1}, \end{array}$$

where *t*_2_ is the time of reception and *t*_1_ is the time of transmission.

According to the distance formula between two points in European space, the distance *D* between GPS user receiver and GPS satellite can be obtained as follows.

(2) $$\begin{array}{c} D=\sqrt{{\left(x_{i}-x\right)}^{2}+{\left(y_{i}-y\right)}^{2}+{\left(z_{2}-z\right)}^{2}}, \end{array}$$

where *D* represents the distance between GPS user receiver and GPS satellite, which is also called observation; (*x*_*i*_, *y*_*i*_, *z*_*i*_) represents the orbit coordinates of each satellite, and (*x*, *y*, *z*) represents the coordinates of GPS user receiver.

Assuming that the difference between the instantaneous time when the GPS receiver receives the GPS satellite signal and the time of the GPS satellite positioning and navigation system is a fixed value Δ*t*, the formula should be modified as follows.

(3) $$\begin{array}{c} D=\sqrt{{\left(x_{i}-x\right)}^{2}+{\left(y_{i}-y\right)}^{2}+{\left(z_{2}-z\right)}^{2}}+\Delta t\times C, \end{array}$$

where *C* is a constant, that is, the propagation speed of GPS satellite signals in space, which is generally set as the speed of light; Δ*t* represents the clock difference between GPS satellite and GPS user receiver, Δ*t*=*t* − *t*_*i*_. The position information of GPS user receiver can be obtained by solving two similar equations.

(4) $$\begin{array}{c} \left\{\begin{array}{c} D_{1}=\sqrt{{\left(x_{1}-x\right)}^{2}+{\left(y_{1}-y\right)}^{2}+{\left(z_{1}-z\right)}^{2}}+\left(t-t_{1}\right)\times C,\\ D_{2}=\sqrt{{\left(x_{2}-x\right)}^{2}+{\left(y_{2}-y\right)}^{2}+{\left(z_{1}-z\right)}^{2}}+\left(t-t_{2}\right)\times C,\\ D_{3}=\sqrt{{\left(x_{3}-x\right)}^{2}+{\left(y_{3}-y\right)}^{2}+{\left(z_{3}-z\right)}^{2}}+\left(t-t_{3}\right)\times C,\\ D_{4}=\sqrt{{\left(x_{4}-x\right)}^{2}+{\left(y_{4}-y\right)}^{2}+{\left(z_{4}-z\right)}^{2}}+\left(t-t_{4}\right)\times C, \end{array}\right. \end{array}$$

where *D*_1_ ~ *D*_4_ represent the distance between GPS satellite and GPS user receiver; (*x*_*i*_, *y*_*i*_, *z*_*i*_) is the satellite orbit coordinates; and *t*_1_ − *t*_4_ is the satellite GPS and GPS user receiver clock difference.

### 3.2. GPS Measurement Advantage

The nonrenewability of land determines the importance of rational use of land. Land use survey is the main means to understand the characteristics and laws of land resources and to master the quantity, quality, and distribution pattern of land resources, and is the basic work to carry out land resources research. Three-dimensional coordinate data are measured by GPS. In practical application, two-dimensional images are generally used to display farmland geographic information [25]. Because the requirement of measurement accuracy is far lower than that of professional surveying and mapping, and only the local area is measured, the simplified method is adopted for data calculation.

If the radius of the earth is taken, the taboo coordinate information data points of any point (*X*, *Y*) are converted into coordinate points (*x*, *y*) in plane coordinates.

(5) $$\begin{array}{c} x=\frac{2\pi \text{RX}}{360},\\ y=\frac{2\pi \text{RY}}{360}. \end{array}$$

In the above formula, *R* represents the radius of the earth, *x* represents the longitude/m, and *y*represents the latitude/m.

Then, the distance between any two points *P*1(*x*, *y*) and *P*2(*x*, *y*) is given by

(6) $$\begin{array}{c} L=\sqrt{{\left(x_{2}-y_{1}\right)}^{2}}. \end{array}$$

At the *Y* degree of the earth's surface, the square area with longitude difference and latitude difference of one degree each is given by

(7) $$\begin{array}{c} A=\frac{2\pi R}{360}\times \frac{2\pi R\times \;\cos\;Y}{360}. \end{array}$$

For the polygon obtained in the measurement, assuming that it is composed of *n* points, the calculation formula of the surrounding area is as follows:

(8) $$\begin{array}{c} S=\left|\sum_{i=1}^{n}\frac{1}{2}\left(x_{i+1}-x_{i}\right)\right|,\\ x_{n+1}=x_{1}=0,\\ y_{n+1}=y_{1}=0. \end{array}$$

The absolute value of the correction number (*V*^Δ*x*^, *V*^Δ*y*^, *V*^Δ*z*^) of the baseline shall meet the requirements of the following formula:

(9) $$\begin{array}{c} V^{\Delta x}\leq 3,dV^{\Delta y}\leq 3,dV^{\Delta z}\leq 3. \end{array}$$

In which $\sigma =\sqrt{a^{2}+{\left(b\;d\right)}^{2}}$; *a* is the fixed error of the receiver, *b* is the proportional error coefficient, and *d* is the distance (*km*) between adjacent points.

The difference (*dV*^Δ*x*^, *dV*^Δ*y*^, *dV*^Δ*z*^) between the vector correction number of the baseline and the corresponding correction number of the baseline of the same name of the unconstrained adjustment result after gross errors are removed shall meet the requirements of the following formula:

(10) $$\begin{array}{c} dV^{\Delta x}\leq 2;dV^{\Delta y}\leq 2;dV^{\Delta z}\leq 2. \end{array}$$

GPS technology can quickly locate spatial data. RS technology can use aerial photographs, satellite photographs, and other image data provided by aerospace and aerial remote sensing to accurately locate and quantify land blocks, and visually interpret the characteristics of ground objects and the current situation of resources [26]. Since the application of GPS positioning technology in surveying engineering, it has the advantages of high automation, all-weather operation, and high precision. The specific performance is explained as follows.

#### 3.2.1. Flexible Point Selection

Different from traditional control survey, GPS positioning technology has low requirements for intervisibility between points. Unless there are special requirements, intervisibility is generally not required, and there are few flexible restrictions on point selection. It reduces the requirement of point network structure.

#### 3.2.2. Being Weather-Independent

GPS positioning can basically realize all-weather operation and normal operation under normal weather conditions.

#### 3.2.3. High Degree of Automation and Convenient Operation

When the operator carries the instrument for operation, after placing the instrument and opening it, he only needs to measure the height of the instrument and monitor the working state of the instrument. The instrument can automatically receive the GPS satellite signal, thus reducing the difficulty of operation and effectively improving the work efficiency.

#### 3.2.4. High Accuracy

When the distance is ≥1000 km, the relative positioning accuracy reaches 10–8; when the distance is 50∼500 km, the relative positioning accuracy reaches 10–6–10–7; and when the distance is ≤50 km, the relative positioning accuracy reaches 10–6. On the contrary, there is no need to build survey targets.

Remote sensing and global positioning systems are primarily used in the application of GIS technology in land use planning and management to obtain spatial data. On this foundation, a land use dynamic remote sensing monitoring system and a land use change management information system are set up to support the creation and revision of planning, the creation of annual land use plans, the preliminary review of construction project land, the review of land use planning for approval, and the administration of land development and consolidation projects. Inspection by law enforcement and monitoring of planning and implementation [27, 28] is constrained by the following: first, satellite circumstances—the working time is limited by the satellite signal being blocked for an extended period of time in high mountains, dense forests, and urban high-rise areas. This problem can be solved by choosing the working time; and second, the data link transmission, which is impeded and limited, and the operation radius, which is shorter than the nominal distance.

## 4. Realization of Surveying and Mapping Method of Landownership

### 4.1. Application and Analysis of GPS Survey Technology in Land Right Confirmation Survey

For the application of GPS technology in land right confirmation survey, in order to ensure the accuracy of survey results, it is necessary to select an area with an open field of vision and no cover in the air, so as to facilitate the transmission of survey information between mobile stations and reference stations through GPS satellites. The preparation of measurement related data, including data creation, import, and export. The different requirements of the operation require us to make targeted formulation and reasonable selection. Only the early work is well selected, good data analysis is carried out, and input is made, which plays a good guarantee for the later work. In the process of rural land cadastral survey, if we want to improve the accuracy of mapping, we often choose the fourth-class control point as the reference point to lead the control point to the required rural area. Since most of the observation data of real-time dynamic measurement are independent observation values, there is no way to calculate the test value with high accuracy through the data. Therefore, we will choose to use the form of repeated observation and total station traverse retest to ensure the accuracy of the final measurement result. GPS-RTK technology is applicable to large survey radius. Plain areas can meet the survey requirements of 18 km, while the operation radius in areas with complex terrain can reach about 9 km, and the survey accuracy can meet the survey requirements of a land planning topographic map. It is necessary to try to stay away from places with strong interferences, such as radio signal transmission towers and high-voltage lines. Because the radio signal will strongly interfere with the GPS satellite signal, resulting in inaccurate data. The required instruments and equipment shall be selected according to the technical requirements and operating environment. Generally, dual-frequency receiver and multifrequency receiver shall be selected. Compared with other receiving equipment, they have higher reliability and stability to ensure that the measurement results are highly representative. After the benchmark station and mobile station are installed, professionals can be organized to conduct field survey.

During the measurement process, the number of operation teams must be selected according to the size of the actual measurement area, and the operators are required to operate in strict accordance with the measurement specifications. The stability of the basic structure of the reference station shall be ensured as far as possible, which can operate stably for a long time and facilitate the implementation of various testing operations. Besides, it shall be convenient to install various instruments and equipment around the station site, and the field of vision shall be expanded with good information transmission conditions. In the land right confirmation work, satellite images were generally used before. With the development of UAV technology, the images taken by UAV have the advantages of high resolution, good image quality, stable received signal, and so on. They are relatively good data sources. If you choose to use a split receiver, you need to focus on the host antenna connection, host radio connection, and the connection between the radio and the data link transmitting antenna. The use of spatial database is to associate complex parcel spatial data with attribute data, and establish a flexible geospatial database. It is spatial data engine rather than spatial database that operates spatial data. It mainly acts as a bridge between relational database and program. The spatial database engine can not only transfer the spatial data to the database for storage, but also obtain the spatial database. GPS survey technology and total station survey are selected to carry out relevant cadastral survey and carry out detailed field survey for all villages. GPS is generally used in the encrypted survey of the mapping control points, and the total station carries out a detailed survey. The reasonable use of GPS and total station promotes the successful completion of the cadastral survey in a short time, and also improves the accuracy of survey. Therefore, we need to encode the data of spatial database and use a unified format to build a complete database. Whether in plane or vertical aspects, attribute data and spatial attribute data need to be nested. The reason why we use spatial database is to enable the landownership confirmation system to efficiently query spatial data, display maps, and operate layers and other functions. It is of great significance to improve the efficiency of land resources development and management. In order to give full play to its advantages, it is necessary to take measures to control each link based on the technical principles and the key points of technical application, so as to reduce the interference of various factors and improve the accuracy of measurement data.

### 4.2. Experimental Results and Analysis

There are three types of research regional data: statistical data, remote sensing data, and spatial data. Statistical data mainly include the resident population and self-employed export volume of towns and streets in 2021, which comes from the Xiaoshan District Statistical Yearbook. For the goal of minimum planning cost, because the conversion cost between different land use types is difficult to obtain directly, reference [6] proposes to indirectly reflect the conversion cost using the conversion coefficient of land use types. Finally, the conversion cost between different land use types is shown in Table 1.

For the carbon emission expansion target, according to the research on the relationship between different ecosystems and carbon emissions in literature [13, 14], the carbon emission/absorption coefficients of different land use types are obtained, and the carbon emission/absorption matrix caused by the conversion of different land use types is obtained by processing, as shown in Table 2.

The model was trained and tested with 16 groups of data with high data accuracy and consistent change trend. In order to make the training data as much as possible, for 8 items of data in each group, the data of three adjacent quarters are used as a group, and each step length is 1. The model is trained, and the data of one group are selected as the test data group after the model training. According to the above training and testing methods, the prediction results of the prediction model under the conditions of the first set of data sets can be obtained, as shown in Figure 3.

As can be seen from Figure 3, under the condition that the development trend of training data is stable, the predicted value of this method is roughly consistent with the true value curve, and the normalized numerical error is basically within the range of 0.2, so the prediction effect is ideal.

Then, under the condition of the second data set, the prediction results of the prediction model of this method are shown in Figure 4.

As shown in Figure 4, when the training set data fluctuate, the prediction error of the prediction model of this method increases slightly, but the overall accuracy of the result remains at a high level, and the normalized error can basically be controlled within 0.3.

Under different multiobjective systems, the results of land use optimization are compared with the land use structure before optimization, as shown in Table 3.

From the comparison between the optimization results under different multiobjective systems and those before optimization, it can be seen that, on the whole, the proportion of cultivated land is reduced, and the proportion of forest land and construction land is increased. In addition, the proportion of unused land is also reduced, and the land utilization rate is improved. Compared with *M*1, the proportion of cultivated land in *M*2 is smaller, while the proportion of forest land and construction land increases. The proportion of *M*3 forest land has decreased. Therefore, it is considered that in the expansion target, the ecological service value plays a major role, while the carbon emission plays a secondary role. From the difference of *M*3, it can be seen that the carbon emission target has a certain inhibitory effect on the ecological service value target.

In this experiment, reference [7], reference [12], and this method are used to test the classification accuracy of grassland, cultivated land, and forest land. The experimental results are shown in Figures 5–7.

From Figures 5–7, it can be seen that different classification methods have different classification accuracy for different land types. Among the three algorithms, the method in document [7] does not clearly distinguish between forest land and grassland in the classification of green land, i.e., grassland, cultivated land, and forest land. The average accuracy of forest land classification is 58.69%, grassland classification is 55.12%, and cultivated land classification is 70.23%. The method in reference [12] does not clearly distinguish between forest land and grassland. The average accuracy of forest land classification is 73.14%, grassland classification is 65.54%, and cultivated land classification is 78.43%. The classification accuracy of this method is relatively high, including 88.45% for forest land, 85.25% for grassland, and 90.53% for cultivated land. Through the comparison of classification accuracy of grassland, cultivated land, and forest land, it can be seen that literature [7] and literature [12] are not as effective as this method in distinguishing small differences between ground objects, because these three ground types are particularly similar in spectral characteristics.

## 5. Conclusions

With regard to measuring landownership, GPS technology measurement offers a number of benefits over more conventional measurement techniques, including quick observation times, all-weather operation, and ease of use. Additionally, GPS technology has a measurement range that is essentially greater than 10 km, which significantly increases measurement accuracy. The surveying and mapping techniques used to determine landownership are examined in this paper using GPS technology. With respect to various land types, various classification methods have varying degrees of classification accuracy. The average classification accuracy for woodland is 58.69 percent among the three algorithms, and the method in reference [7] does not make it clear enough to differentiate it from grassland. The average accuracy of woodland classification in reference [12] is 73.14 percent, but it is not clear how to tell woodland from grassland. Although the methods used in this paper have a relatively high classification accuracy, woodland has the highest classification accuracy at 88.45%. It can be seen that literature [7] and literature [12] are not as accurate as the method in this paper in identifying minute differences between ground objects. This is because the classification accuracy of forest land is not as high. The advancement and use of GPS technology has significantly raised the working standard for rural collective land certification and registration. This improvement is primarily seen in the measurement's accuracy and convenience. The GPS technology survey also has low requirements for the field of vision, which somewhat lowers the requirements of the working environment. The data's high accuracy also fully satisfies the criteria for the accuracy of landownership surveys.

## Figures and Tables

**Figure 1:** Composition model of GPS satellite signal.

**Figure 2:** Principle of GPS satellite positioning.

**Figure 3:** Change trend of predicted values of the first group of data.

**Figure 4:** Change trend of predicted values of the second group of data.

**Figure 5:** Comparison of grassland classification accuracy between three methods.

**Figure 6:** Comparison of cultivated land classification accuracy between three methods.

**Figure 7:** Comparison of forest land classification accuracy between three methods.

**Table 1:** Land-type conversion factor in minimum planning cost.

	Plough	Lawn	Woodland	Land for construction	Unused land
Plough	0	0.4	0.6	0.2	—
Lawn	0.2	0	0.7	0.1	—
Woodland	0.8	0.5	0	0.8	—
Land for construction	—	—	—	0	—
Unused land	0.2	0.8	0.6	0.2	0

**Table 2:** Land conversion factors in carbon emission targets.

	Plough	Woodland	Grassland	Land for construction
Cultivated land	0.5016	0.2681	0.4823	0.7681
Grassland	0.7317	0.2698	0.7301	1.0012
Woodland	0.5175	0.2701	0.4997	0.7704
Land used for building	0.2317	0.0000	0.2305	0.7698

**Table 3:** Comparison of land use structure after optimization of different multiobjective systems.

		Cultivated land, %	Woodland, %	Grassland, %	Construction land, %	Unused land, %
	2020	40.35	16.11	0.03	42.42	0.52
*M*1	After optimization	37.05	16.75	0.04	45.48	0.11
	Increase	−3.2	0.65	−0.02	3.07	−0.42
*M*2	After optimization	36.75	17.02	0.01	45.25	0.07
	Increase	−3.7	0.92	−0.01	3.14	−0.44
*M*3	After optimization	37.87	18.81	0.03	42.46	0.24
	Increase	−2.47	2.8	0	0.05	−0.27

## Data Availability

The data used to support the findings of this study are available from the author upon request.
